# Functional Conservation of the *Drosophila gooseberry* Gene and Its Evolutionary Alleles

**DOI:** 10.1371/journal.pone.0030980

**Published:** 2012-01-23

**Authors:** Wei Liu, Lei Xue

**Affiliations:** 1 College of Veterinary Medicine, Northwest Agriculture & Forest University, Yangling, Shaanxi, China; 2 School of Life Science and Technology, Tongji University, Shanghai, China; 3 Institute for Molecular Biology, University of Zürich, Zurich, Switzerland; National Cancer Institute, United States of America

## Abstract

The *Drosophila Pax* gene *gooseberry* (*gsb*) is required for development of the larval cuticle and CNS, survival to adulthood, and male fertility. These functions can be rescued in *gsb* mutants by two *gsb* evolutionary alleles, *gsb-*Prd and *gsb-*Pax3, which express the *Drosophila* Paired and mouse Pax3 proteins under the control of *gooseberry cis*-regulatory region. Therefore, both Paired and Pax3 proteins have conserved all the Gsb functions that are required for survival of embryos to fertile adults, despite the divergent primary sequences in their C-terminal halves. As *gsb-*Prd and *gsb-*Pax3 uncover a *gsb* function involved in male fertility, construction of evolutionary alleles may provide a powerful strategy to dissect hitherto unknown gene functions. Our results provide further evidence for the essential role of *cis*-regulatory regions in the functional diversification of duplicated genes during evolution.

## Introduction

During early *Drosophila* embryogenesis, the antero-posterior axis is progressively defined by the activities of four classes of segmentation genes: maternal coordinate genes, zygotic gap genes, pair-rule genes, and segment-polarity genes [1]–[4]. In addition to their roles in patterning the embryonic epidermis, many segmentation genes participate in other developmental programs like neurogenesis [5], myogenesis [6], and development of imaginal discs [7].

The *Drosophila gooseberry* (*gsb*) gene, initially identified as a member of the segment-polarity gene class [1], is required after germ band extension to maintain the ventral epidermal expression of *wingless* (*wg*), which suppresses ubiquitous denticle formation, through a *wg*-*gsb* autoregulatory loop [8]. In the central nervous system (CNS), *gsb* is essential for the activation of *gooseberry neuro* (*gsbn*) in a segmentally repeated pattern [9], for the differentiation of certain neuroblasts, and for the formation of the posterior commissure in each segment [10]–[14]. Since all known *gsb* mutant alleles are embryonic lethal [11], possible postembryonic functions of *gsb* remain largely unknown. Recently, *gsb* has been found to sustained expression of synaptic homeostasis, indicating the existence of postembryonic functions [15].

*gsb* encodes a transcription factor including two DNA binding domains in its N-terminal moiety, a paired-domain and a *prd*-type homeodomain [16]–[18]. Both domains are highly conserved in the N-terminal halves of the *Drosophila* Paired (Prd) and mouse Pax3 proteins, whose C-terminal halves, however, seem unrelated in their primary sequences to the C-terminal portion of Gsb [17], [19]. *prd* is a member of the pair-rule gene class, specifying position along the antero-posterior axis with a double-segment periodicity and regulating the expression of segment-polarity genes [20]. The *Pax3* gene, a mutation in which is responsible for the *Splotch* phenotype in mice [21] and Waardenburg's syndrome I in humans [22], [23], plays a pivotal role in myogenesis [24].

Despite their divergent developmental functions, Gsb and Pax3 proteins are able to substitute for most functions of Prd when expressed under the control of the complete *prd cis*-regulatory region in *prd*-Gsb and *prd*-Pax3 transgenes [25]. While *prd*-Pax3 is able to rescue the cuticular phenotype of *prd* mutants, *prd*-Gsb can further rescue *prd* mutants to adulthood [25], though the rescued males show reduced accessory glands and are sterile [26]. Taken together, these results indicate that Gsb, and Pax3 proteins have retained most functions of Prd despite their highly diverged C-terminal halves and further point to the *cis*-regulatory region as an important determinant for the functional diversification of these three genes. However, these experiments left unanswered the question of whether Prd and Pax3 proteins could substitute for the normal functions of Gsb.

To address this question, we produced two “evolutionary alleles” [25] of *gsb*, namely *gsb-*Prd and *gsb-*Pax3, which express Prd or Pax3 proteins under the control of the complete *gsb cis*-regulatory region. We show that both transgenes are able to rescue *gsb* mutants to fertile adults, albeit at reduced efficiencies, which suggests that both Prd and Pax3 proteins have conserved all normal functions of Gsb. We conclude that the divergent functions of *gsb*, *prd*, and *Pax3* genes are predominantly determined by their different *cis*-regulatory regions and are further modified by their protein coding regions. These results provide additional evidence to our previous model that the acquisition of different *cis*-regulatory elements is the primary mechanism in the evolution of new functions [25]. Since some of the rescued males are sterile, *gsb* is important for male fertility. This discovery of a male fertility function of *gsb* suggests that the construction of “evolutionary alleles” may serve as a powerful tool to reveal the hitherto unknown functions of a gene.

## Results

### Characterization of two hypomorphic *gsb* alleles

The *gsb* gene was initially uncovered by two large deficiencies, *Df(2R)IIX62* and *Df(2R)Kr^SB1^*, obtained in a screen for embryonic segmentation mutants [1]. Transheterozygotes of the two deficiencies have lost at least two genes in addition to *gsb* (**Figure 1A**). Their cuticle shows a strong segment-polarity phenotype (Fig. 2C), which is indistinguishable from that of homozygous *Df(2R)IIX62* embryos (**Figure 2B**) [1].

**Figure 1:** Locus of the *gsb* gene. (**A**) *gsb* mutant alleles. The two deficiencies, *Df(2R)IIX62* and *Df(2R)SB1*, as well as the two hypomorphic alleles, *gsb525* and *gsbP1155*, are depicted. Neighboring genes uncovered by *Df(2R)IIX62*, *zip*, *uzip*, *CG3441*, and *gsbn* upstream of *gsb*, *gol* and *dTKR* downstream of *gsb*, and their direction of transcription are indicated (the rigth telomere of the second chromosome is to the right). Exons are marked by black boxes in the enlarged portion of (**A**) and also in (**B**). (**B**) Map of *gsb0-*525 abd *gsb0*-ΔHC transgenes. Both transgenes contain the upstream epidermis enhancers of *gsb*, GEE and GLE (**Fig. 1A**; Li et al., 1993), the *gsb* promoter, and the entire 3′ UTR of *gsb*. In *gsb0*-ΔHC, 519 bp of coding region between the *gsb525* mutation and a *SacII* site are deleted, resulting in a shift of the open reading frame after the *gsb525* nonsense mutation. (**C**) Sequence surrounding the *gsbP1155* insertion site. The negative numbers refer to nucleotides upstream of the transcription start site. The eight nucleotides, duplicated during insertion of the P-element, are underlined.

**Figure 2:** Cuticular phenotypes of *gsb* mutants. (**A**) *Df(2R)IIX62/CyO*, (**B**) *Df(2R)IIX62*, (**C**) *Df(2R)IIX62/Df(2R)KrSB1*, (**D**) *Df(2R)IIX62/gsb525*, (**E**) *gsb525*, (**F**) *gsbP1155*, (**G**) *Df(2R)IIX62*; *gsb0*-525 (**H**) *Df(2R)IIX62*; *gsb0*-ΔHC. Note in strong *gsb* mutants (**B**, **C**), the ventral naked cuticle region of each segment is transformed into denticle belt, generating an overall denticle pattern, which is in contrast to wild-type (**A**). Scale bar: 50 um.

Two alleles affecting only the *gsb* gene were identified late, including a point mutation, *gsb^525^*, and a P-element insertion, *gsb^P1155^* [11]. In *gsb^525^*, the codon of the first amino acid of the homeodomain is mutated to a TAA stop codon. In *gsb^525^* embryos, the *gsb* mRNA level is much reduced by stage 11, presumably because *gsb* activity depends on the *wg-gsb* autoregulatory loop [8], and no Gsb protein is detected by immunostaining, while the protein product of the Gsb target, Gsbn, is barely detectable. The fact that *gsb^525^/Df(2R)IIX62* embryos exhibit only a weak cuticular phenotype (**Figure 2D**), while that of *gsb^525^* embryos (**Figure 2E**) is nearly wild-type (**Figure 2A**) implies that *gsb^525^* is not a null allele [11]. Its hypomorphic nature might be explained in two not mutually exclusive ways: the cuticular function of *gsb* is provided either by a Gsb^525^ protein truncated before the homeodomain but including the entire paired domain, or by undetectable levels of wild-type Gsb protein generated by a low probability of read-through at the *ochre* nonsense mutation. To elucidate this question, we prepared two rescue constructs. *gsb0-*525 contains the same mutation as *gsb^525^*, whereas *gsb0-*ΔHC encodes only the truncated Gsb^525^ protein (**Figure 1B**). Both of these two constructs are under the control of the *gsb* upstream region including the *gsb* cuticle enhancers GEE and GLE [26]. Evidently, only *gsb0*-525 can rescue the cuticle phenotype (**Figure 2G**), whereas *gsb0-*ΔHC cannot (**Figure 2H**). This demonstrates that in *gsb^525^* embryos an undetectable level of wild-type Gsb protein is produced that is nearly enough to rescue the cuticular function of *gsb*.

*gsb^P1155^* is also an interesting allele. It is an insertion of a P element located only 54 bp upstream of the *gsb* transcription start site (**Figure 1C**). This P-element insertion leads to largely reduced *gsb* mRNA and protein levels in homozygous embryos. While these mutants show a wild-type cuticular phenotype (**Figure 2F**) and only mild CNS defects [11], we observed a strongly reduced expression of *gsbn* (data not shown). It follows that *gsb^P1155^* is a weaker allele than *gsb^525^*.

### Generation of *gsb-*Prd and *gsb-*Pax3 transgenic flies

Previous work demonstrated that a *gsb* rescue construct, *gsb-res*, was able to perform all the known *gsb* functions and rescue *gsb* mutants to adulthood [9], [11], which suggests that all essential *gsb* enhancer elements are included in this *gsb* transgene (**Figure 3**). To examine whether and to what extent the Prd and Pax3 proteins are able to substitute for the normal functions of Gsb, two rescue constructs, namely *gsb-*Prd and *gsb-*Pax3, were obtained by replacing the *gsb* coding region in *gsb-res* by that of *prd* and *Pax3*, respectively (**Figure 3**). Transgenic files were generated by P-element-mediated transformation in the *Drosophila* germlines [31]. Several independent lines were obtained for each construct. Only transgenic lines that were homozygous viable were selected for further investigation.

**Figure 3:** Map of *gsb-res*, *gsb-*Prd and *gsb-*Pax3 transgenes. The *gsb-res* transgene corresponds to the enlarged 20-kb genomic fragment in **Fig. 1A**, which includes the *gsb* transcribed region as well as adjacent 14-kb upstream and 3-kb downstream sequences [9]. The upstream sequence also contains the 5′ portion of the *gsbn* up to part of the third exon. In *gsb*-Prd and *gsb*-Pax3 transgenes, the *gsb* coding region (except of a small region encoding the C-terminus) is replaced by *prd* and *Pax3* cDNAs, while upstream and downstream regions are retained. The *gsb* intron is also retained by inserting it between sequences of the *gsb* and *prd* or *Pax3* leaders. Coding regions are indicated as black boxes except for the paired-domain (PD) and the *prd*-type homeodomain (HD) which are hatched. The *gsb* and *gsbn* introns are indicated as open boxes. The transcription start of *gsb* is marked by 0, and poly(A) addition signals AATAAA are indicated.

It has been previously shown that in wild-type embryos, Gsb protein is initially expressed during blastoderm at the end of cellularization in eight stripes in every other segment, which correspond to the odd-numbered Gsb stripes [9]. At gastrulation, the even-numbered Gsb stripes emerge between the odd-numbered stripes to generate a segmentally repeated expression pattern. Toward the end of germ band extension, Gsb protein reaches its highest levels in the ectoderm and becomes laterally restricted to the neuroectodermal region (**Figure 4A**). As expected, in *gsb-*Prd and *gsb-*Pax3 embryos, the Prd protein (**Figure 4B**) and *Pax3* mRNA (**Figure 4C**) are expressed in patterns that are indistinguishable from that of endogenous Gsb protein (**Figure 4A**). At this time of development the endogenous Prd protein is barely detectable in the epidermis [27].

**Figure 4:** Expression of Gsb and Prd proteins and *Pax3* mRNA under control of the *gsb cis*-regulatory region. Expression of Gsb protein in wild-type embryos (*ry^506^*; **A**), of Prd protein in transgenic *gsb*-Prd embryos (**B**), and of *Pax3* mRNA in transgenic *gsb*-Pax3 embryos (**C**) at the extended germ band stage. Wild-type embryos were stained with anti-Gsb antiserum and transgenic embryos, collected from homozygous *gsb*-Prd or *gsb*-Pax3 stocks, were stained with anti-Prd antiserum or hybridized *in situ* with digoxigenin-labeled *Pax3* cDNA. Unfolded embryos are shown and oriented with their anterior to the left. Scale bar: 100 um.

### Rescue of *gsb* target gene expression by *gsb-*Prd and *gsb-*Pax3

Previous work has shown that Gsb is required to maintain late *wg* expression in the ventral epidermis through a *wg-gsb* autoregulatory loop [8]. In homozygous *Df(2R)IIX62* embryos, Wg starts to decay in the ventral epidermis after 6 hours [8] and is no longer detectable at stage 13 (**Figure 5B**), while it remains expressed in wild-type embryos (**Figure 5A**). By introducing *gsb-*Prd or *gsb-*Pax3 transgenes into such *gsb* mutant embryos, the Wg expression pattern is fully rescued by one copy of either transgene (**Figure 5C, D**).

**Figure 5:** Rescue of Wg and Gsbn expression in *gsb* mutant embryos by *gsb*-Prd and *gsb*-Pax3 transgenes. Expression of Wg (**A–D**) and Gsbn (**E–H**) proteins in wild-type (**A, E**), homozygous *Df(2R)IIX62* (**B–D**) or transheterozygous *Df(2R)IIX62/gsb525* (**F–H**) *gsb* mutant embryos carrying no (**B, F**), one copy of the *gsb*-Prd (**C, G**) or *gsb*-Pax3 (**D, H**) transgene. Embryos at stage 13 (**A–D**) or stage 10 (**E–H**) are oriented with their anterior to the left and dorsal side up. Embryos were collected from crosses between *Df(2R)IIX62/*CyO, *hb*-LacZ; *gsb*-Prd/+ or *Df(2R)IIX62/CyO*, *hb-*LacZ; *gsb-*Pax3/+ males and *Df(2R)IIX62/CyO*, *hb-*LacZ (**A–D**) or *gsb525/CyO*, *hb-*LacZ females (**E–H**), and double stained for ß-galactosidase and or Gsbn protein with rabbit antiserum against ß-galactosidase and anti-Wg monoclonal antibodies or rabbit anti-Gsbn antiserum. Embryos stained with ß-galactosidase have at least one copy of wild-type *gsb* allele and were used as control (**A**, **E**). One quarter of the embryos did not stain for ß-galactosidase. Half of these embryos did not express Wg in the ventral epidermis and Gsbn in the CNS as expected for *gsb* mutants. The other half displayed rescued expression patterns, which suggested the presence of the transgenes. Scale bar: 100 um.

Beginning with stage 9, Gsb is expressed in delaminating neuroblasts, where it is required for the activation of *gsbn* [9]. This is apparent from a complete loss of Gsbn expression in *Df(2R)IIX62/gsb^525^* embryos at the extended germ band stage (**Figure 5F**), while Gsbn expression is strongly expressed in the CNS of wild-type embryos at this stage (**Figure 5E**). Gsbn expression in such mutants are rescued by *gsb-*Prd or *gsb-*Pax3 transgene, respectively (**Figure 5G, H**). Taken together, these results demonstrate that Prd and Pax3 proteins can substitute for Gsb function in the transcriptional activation of two essential target genes.

### Rescue of *gsb^-^* cuticular phenotype by *gsb-*Prd and *gsb-*Pax3

One conspicuous feature of the *Drosophila* larva is the metameric ventral cuticular pattern, which crucially depends in each segment on the products of the segment-polarity genes. Embryos lacking *gsb* function exhibit a segment-polarity cuticle defect [1], which consists of mirror image duplications of denticle belts into the posterior portions of each segment where naked cuticle would develop in wild-type embryos (compare **Figure 6A, B**). This phenotype is caused by the loss of late Wg expression, which is required to repress the ubiquitous denticle formation in the ventral epidermis [8]. Consistent with the result that both *gsb-*Prd and *gsb-*Pax3 can rescue the late Wg expression in *gsb* mutants, both transgenes are able to fully rescue the cuticular phenotype of homozygous *Df(2R)IIX62* embryos when present as a single copy (**Figure 6C, D**). It follows that Prd and Pax3 proteins are able to perform the cuticular function of Gsb.

**Figure 6:** Rescue of the cuticular phenotype of gsb mutant embryos by gsb-Prd and gsb-Pax3 transgenes. Ventral view of cuticle preparations of wild-type (*ry^506^*; **A**) and homozygous *Df(2R)IIX62* embryos without (**B**) and with one copy of the gsb-Prd (**C**) or gsb-Pax3 transgene (**D**) are shown under dark-field illumination (anterior is up). Wild-type and *gsb* mutant embryos were collected from the *Df(2R)IIX62/SM1* stock, while gsb mutant embryos carrying one copy of the transgenes were collected from crosses between *Df(2R)IIX62/SM1*; *gsb-Prd* or *Df(2R)IIX62/SM1; gsb-Pax3* males and *Df(2R)IIX62/SM1* females. *gsb* mutants were distinguished from wild type by the presence of the zip phenotype, a deformed head structure resulting from the deletion of the zip gene, which is uncovered by *Df(2R)IIX62* [30]. Scale bar: 50 um.

### Rescue of *gsb^-^* CNS phenotype by *gsb-*Prd and *gsb-*Pax3

In addition to its function in patterning the epidermis, *gsb* plays an important role in the development of the embryonic CNS [9]–[12]. Most prominently, posterior commissures (**Figure 7A**) are missing or reduced in each segment of *Df(2R)IIX62*/*gsb^525^* embryos (**Figure 7B**). This CNS phenotype can be fully rescued by one copy of the *gsb-*Prd (**Figure 7C**) or *gsb-*Pax3 transgene (**Figure 7D**), which indicates that Prd and Pax3 proteins are able to replace the Gsb function in the CNS.

**Figure 7:** Rescue of the CNS phenotype of *gsb* mutant embryos by *gsb*-Prd and *gsb*-Pax3 transgenes. Patterns of longitudinal and commissural axons in the CNS of wild-type (*ry^506^*; **A**) and *Df(2R)IIX62/gsb525* embryos without (**B**) and with one copy of the *gsb*-Prd (**C**) or *gsb*-Pax3 transgene (**D**). Embryos at stage 15 were collected from crosses between *Df(2R)IIX62/CyO*, *hb-*LacZ; *gsb*-Prd/+ or *Df(2R)IIX62/CyO*, *hb-*LacZ; *gsb-*Pax3/+ males and *gsb525/CyO*, *hb-*LacZ females, and double stained with rabbit antiserum against ß-galactosidase and monoclonal antibody BP102. One quarter of the embryos did not stain for ß-galactosidase as expected. Half of these embryos have missing or reduced posterior commissures as expected for *gsb* mutants, the other half displays fully rescued commissural patterns as in wild-type embryos. Scale bar: 10 um.

### Rescue of *gsb* mutants to adulthood by *gsb-*Prd and *gsb-*Pax3

To test if Prd and Pax3 proteins are able to substitute for all Gsb functions, we tested the ability of *gsb-*Prd and *gsb-*Pax3 transgenes to rescue *gsb* mutants to adulthood. For this purpose, a deficiency, *Df(2R)IIX62*, and two strong alleles of *gsb*, *gsb^525^* and *gsb^P1155^*, were used. Homozygous or heterozygous combinations of these three alleles are lethal during embryogenesis, which shows that *gsb* is required for postembryonic viability. Although rescue efficiencies are less than half of that of *gsb-res*, one copy of *gsb-*Prd or *gsb-*Pax3 is able to rescue about a quarter of *Df(2R)IIX62/gsb^525^* embryos to adulthood (**Table 1**). For all three transgenes, two copies result in 50% higher rescue efficiencies than one copy (**Table 1**), which suggests that at least one *gsb* function required for the viability is dosage dependent. Consistent with this interpretation, one copy of the transgenes is able to rescue a much higher proportion of *Df(2R)IIX62/gsb^P1155^* or *gsb^525^/gsb^P1155^* embryos to adulthood (**Table 1**). Therefore, both Prd and Pax3 proteins are able to substitute for all Gsb functions required for survival to adulthood, albeit at lower efficiencies.

**Table 1:** Rescue of *gsb* mutant embryos to viable adults by *gsb*-Prd and *gsb*-Pax3 transgenes.

	*gsb-res* (%)		*gsb-*Prd (%)		*gsb-*Pax3 (%)	
	1 copy	2 copies	1 copy	2 copies	1 copy	2 copies
*Df(2R)IIX62/gsb^525^*	62 (238/385)	96 (194/203)	21 (90/429)	31 (104/339)	27 (88/326)	**41 (96/234)**
*Df(2R)IIX62/gsb^P1155^*	86 (607/707)	nd	51 (144/284)	nd	74 (192/260)	**nd**
***gsb^525^/gsb^P1155^***	**99 (344/346)**	**nd**	**61 (230/376)**	**nd**	**77 (226/293)**	**nd**

Percentage of rescued *gsb^-^* flies harboring one or two copies of *gsb-res*, *gsb-*Prd or *gsb-Pax3* transgenes (actual numbers of rescued flies per total number of expected *gsb* mutants are given in parentheses). *Df(2R)IIX62/gsb^525^* flies carrying one or two copies of the transgenes were obtained as offspring from the crosses between *Df(2R)IIX62/SM1*; *P/P* (P stands for the transgenes) males and *gsb^525^/SM1* or *gsb^525^/SM1*; *P/P* females. *Df(2R)IIX62/gsb^P1155^* and *gsb^525^/gsb^P1155^* flies carrying one copy of the transgenes were obtained from the crosses between *Df(2R)IIX62/SM1*; *P/P* or *gsb^525^/SM1*; *P/P* males and *gsb^P1155^/SM1* females. nd, not determined.

### *gsb* is required for male fertility

Since all known *gsb* mutant alleles are lethal during embryogenesis [1], [9], [11], the adult functions of *gsb* remain unknown. Interestingly, most of the *Df(2R)IIX62/gsb^525^* males rescued by one copy of *gsb-*Prd or *gsb-*Pax3 are sterile (**Table 2**), while females are fully fertile (data not shown). Therefore, *gsb* is endowed with a function that is essential for male fertility. Two copies of *gsb-*Prd or *gsb-*Pax3 result in significantly enhanced fertilities of *Df(2R)IIX62/gsb^525^* males (**Table 2**), which suggests that this male fertility function is also dosage dependent. Consistent with this explanation, one copy of *gsb-res* rescues fertility in 39% of the *Df(2R)IIX62/gsb^525^* males, while two copies rescue male fertility almost completely (**Table 2**). In addition, one copy of *gsb-*Prd or *gsb-*Pax3 is able to rescue fertility in about half of the *Df(2R)IIX62/gsb^P1155^* males and in three quarters of the *gsb^525^/gsb^P1155^* males (**Table 2**), whereas one copy of *gsb-res* suffices to fully rescue male fertility in these two mutant combinations (**Table 2**). We conclude that *gsb* is required for male fertility, a function for which both Prd and Pax3 proteins are able to substitute.

**Table 2:** Rescue of fertility of *gsb* mutant males by *gsb*-Prd and *gsb*-Pax3 transgenes.

	*gsb-res* (%)		*gsb-*Prd (%)		*gsb-*Pax3 (%)	
	1 copy	2 copies	1 copy	2 copies	1 copy	2 copies
*Df(2R)IIX62/gsb^525^*	39 (36/92)	91 (20/22)	9 (2/23)	30 (6/20)	15 (3/20)	**35 (6/17)**
*Df(2R)IIX62/gsb^P1155^*	92 (90/98)	nd	43 (16/37)	nd	48 (16/33)	**nd**
***gsb^525^/gsb^P1155^***	**95 (74/78)**	**nd**	**77 (23/30)**	**nd**	**75 (21/28)**	**nd**

Percentage of fertile males among *gsb* mutant males that were rescued by one or two copies of *gsb-res*, *gsb*-Prd or *gsb*-Pax3 transgenes (actual numbers of fertile males per total number of rescued males are given in parentheses). Rescued males were obtained from crosses described in legend of table 1 and were placed individually with at least three wild-type virgin females in fresh vials to score fertility. nd, not determined.

## Discussion

### Evolutionary alleles of *gsb*

The *Drosophila gsb* and *prd* and mouse *Pax3* genes encode transcription factors that share in their N-terminal moieties two DNA binding domains, a paired-domain and a *prd*-type homeodomain [16]–[19]. The homology between the N-terminal parts of the three proteins suggests that they were derived from a common ancestor, and thus might have retained some same abilities, despite their divergent C-terminal sequences and apparently distinct developmental functions [32]. Indeed, *gsb-*Prd and *gsb-*Pax3, which express Prd or Pax3 protein under the control of the *gsb cis*-regulatory region, are able to execute all *in vivo* functions of *gsb*, though less efficiently. Hence, both Prd and Pax3 may be considered as leaky mutant proteins of Gsb, whereas *gsb-*Prd and *gsb-*Pax3 are hypomorphic or ‘evolutionary’ alleles of *gsb*, as the coding regions of the three genes have been derived from a common ancestral gene during the course of evolution. These two ‘evolutionary’ alleles are weaker than the weakest previously known *gsb* allele, *gsb^P1155^*, which generates a normal cuticular pattern but displays a weak CNS phenotype and is homozygous lethal during embryogenesis [11]. As these two new alleles have uncovered the previously unknown function of *gsb* required for male fertility, construction of evolutionary alleles may serve as an additional approach to discover unknown functions of a gene [25].

Although the N-terminal portions of the three proteins are rather conserved, their C-terminal parts have diverged to an extent that no obvious similarity in the primary sequences could be perceived [17], [19]. Thus, it is particularly interesting that both Prd and Pax3 proteins have retained the potential to perform all the normal functions of Gsb, which suggests that all the important functional motives in the C-terminal part of Gsb have been conserved in the C-termini of Prd and Pax3, presumably in the 3-D structures. It follows that the functional diversification of *gsb*, *prd*, and *Pax3* reside in their *cis*-regulatory rather than their divergent C-terminal coding regions. Therefore, our results are consistent with, and add further weight to, the hypothesis that the acquisition of new enhancer elements by a gene plays a dominant role in evolution [25], [26].

### Evolutionary relationship between Gsb, Prd and Pax3 proteins

Our previous work has shown that Pax3 can perform only the cuticle function, but not the viability and male fertility functions of Prd [25], [33]. Here we report that Pax3 is able to substitute for all Gsb functions in promoting embryonic CNS and cuticle development, postembryonic viability, and male fertility. Thus, in terms of functional conservation, Pax3 seems to be more closely related to Gsb than to Prd. It follows that Gsb and Pax3 are functionally also closer to the common ancestor than Prd. As an independent test of this conclusion, it would be interesting to see if Gsb is a better substitute for Pax3 functions than Prd.

In support of this hypothesis, Pax3 resembles Gsb better than Prd in primary sequences. For Gsb and Pax3, but not Prd, share an octapeptide that is located between the paired-domain and the *prd*-type homeodomain [16], [19], [32]. In addition, Prd possesses near its C-terminal end a PRD repeat [34], which is also found in the products of several other genes that are important for early development [34], [35], but not in Gsb and Pax3. Therefore, the common ancestor of Gsb, Prd, and Pax3 probably included, in addition to the paired-domain and the *prd*-type homeodomain, the octapeptide in between. After duplication and separation during the course of evolution, Gsb and Pax3 retained these three motives while Prd lost the octapeptide, but instead, obtained the PRD repeat.

In addition to its embryonic functions, *gsb* is also required for male fertility. This function appears to be dosage dependent, as better rescue efficiencies were achieved by either increasing the copy number of the transgenes or using weaker *gsb* mutant alleles (**Table 2**). Interestingly, *prd* is also required for male fertility, in particular for the development of accessory glands [33], [34]. Since Gsb is able to substitute for all Prd functions that are required for survival to adulthood [25], but not its male fertility function [28], the male fertility function of Prd might have evolved after its separation from Gsb or have been subjected to strong selection during the course of evolution.

### Dosage effect of *Pax* genes

*Pax* genes encode transcription regulators characterized by the presence of the paired-domain [32]. In vertebrates, *Pax* genes exhibit strong dosage effects, as most *Pax* genes are haploinsufficient [36], and overexpression of *Pax6* in mice leads to severe eye abnormalities [37]. In *Drosophila*, *prd* shows haploinsufficiency in an adult segmentation phenotype, and the *prd* evolutionary allele *prd*-Gsb displays strong dosage effects for all *prd* functions required for survival to adulthood [25]. In addition, overexpression of *eyeless*, the *Drosophila* homolog of *Pax6*, results in a small eye phenotype [38]. Here we show that one copy of the *gsb* rescue construct, *gsb-res*, is able to rescue only 62% of the *Df(2R)IIX62/gsb^525^* mutants to adulthood (**Table 1**), of which only 39% of the males are fertile (**Table 2**). However, higher rescue efficiencies were scored in both cases by two copies of the transgene (**Table 1**, **2**), which indicates a dosage dependence of *gsb* functions in promoting viability and male fertility. This interpretation was confirmed by the use of two different combinations of *gsb* mutants, and by two *gsb* evolutionary alleles, *gsb-*Prd and *gsb-*Pax*3* (**Table 1**, **2**). A dosage effect was also reported for *gsb* functions in embryonic cuticle and CNS development, as reflected by differences in penetrance of the cuticle and CNS phenotypes in various combinations of different *gsb* mutant alleles [11]. Since the hypomorphic *gsb* mutants, *gsb^525^* and *gsb^P1155^*, display a normal cuticle but defects in the CNS [11], and one copy of *gsb-res* is able to fully rescue the CNS phenotype but to rescue the viability and male fertility functions only partially (**Table 1** **,** **2**) in *Df(2R)IIX62/gsb^525^* mutants, the cuticle function is least sensitive while the viability and male fertility functions are most sensitive to a decrease in the level of Gsb activity. The incomplete rescue of the viability and male fertility functions in *Df(2R)IIX62/gsb^525^* mutants by one copy of *gsb-res* may result from two effects. First, the deficiency *Df(2R)IIX62*, which deletes, in addition to *gsb*, several other genes including *gsbn* [17], [30], which is downstream of *gsb*, might affect the viability and male fertility. Second, *gsb-res* expresses Gsb protein at a subnormal level [9], [11], which may result from a position effect of the P-element insertion or from the absence of additional *gsb* enhancer element(s) from the transgene.

### The male fertility function of *gsb*

In addition to its embryonic functions, *gsb* is also required for the male fertility. This function appears dosage dependent, for better rescue efficiencies were achieved by either increasing the copy number of the transgenes or using weaker *gsb* mutant alleles (**Table 2**). *gsb* may get involved in male fertility via several means. First, Gsb plays pivotal role in the development of ejaculatory duct that is required for the transfer of accessory gland secretions and sperm to females during copulation. Ejaculatory duct also secretes components of seminal fluid that might be essential for sperm fertility [39]. Second, Gsb is expressed in the secondary cells of adult accessory glands, suggesting a role of Gsb in the regulation of accessory gland secretions that are crucial for the male fertility (33). Third, males heterozygous for *Df(2R)IIX62*, which deletes *gsb* and its downstream gene *gsbn*, behave less aggressive in copulation (data not shown). This phenotype can be rescued by adding one copy of *gsb-res* (data not shown), implying the impaired Gsb-Gsbn pathway is responsible for this behavioral defect. In support of this interpretation, both Gsb and Gsbn are expressed in the leg and antenna imaginal discs (W.L., L.X. and M.N., unpublished observation), suggesting a role of *gsb* and *gsbn* in the development of leg and antenna, both of which have been shown to be important for eliciting proper male sexual behavior [40].

Interestingly, *prd* is also required for male fertility, for *prd* mutant males rescued by two differently modified *prd* transgenes, *prd*-Gsb [25] and *prd*Res [41], are sterile, despite their capabilities to copulate and transfer sperm to females [33]. These males have severely reduced or no accessory glands [33], [41], suggesting *prd* is essential for accessory gland development. Hence, *prd* and *gsb*, though both are required for male fertiltiy, are involved in distinct developmental programs during metamorphosis. Since Gsb is able to substitute for all Prd functions that are required for survival to adulthood [25], but not its male fertility function [33], the male fertility function of Prd might have evolved after its separation from Gsb or have been subjected to strong selection during the course of evolution.

## Materials and Methods

### Plasmid constructions and generation of transgenic flies

Mutations were introduced into *gsb*0-525 and *gsb*0-ΔHC by PCR mutagenesis. Taking pKSpL5-Gsb [27] as template, the following primers were used: gsb-8 (5′-GTC GTC CGG GCT AGC CTT TAT TTC CT-3′), gsb-11 (5′-GGA AAT AAA GGC GAT CGC GGA CG -3′, gsb-12 (5′-CGT CCG CGA TCG CCT TTA TTT CC-3′), T3 primer, and T7 primer. Fragments containing the mutations were cloned into *gsb*-0 [27], the *gsb* complete leader region and intron were also recovered.

The *gsb-*Prd and *gsb-*Pax3 constructs were derived from *gsb-res* [9] in three steps. First, the 1-kb *gsb* intron was obtained as a PCR product with the primer gint1 (5′-GTC TAG AGT AAG CAC CGA CAG ATA GA-3′) and gint2 (5′-GTC TAG ACT GGA AGA ATT AGA GAA ACA-3′), digested with *Xba*I and inserted into the *Spe*I site of pKSpL5-Prd and pKSpL5-Pax3 [27] to generate pKSgint-Prd and pKSgint-Pax3, respectively. Subsequently, the 3.4-kb *Xba*I fragments from pKSgint-Prd and pKSgint-Pax3 were cloned into the *Avr*II site of *gsb*-0 to produce *gsb*-*int*-Prd and *gsb*-*int*-Pax3. Finally, *gsb-*Prd and *gsb-*Pax3 were constructed by replacing the 5.6-kb *Nhe*I-*Xba*I fragment in *gsb-res* with the corresponding fragments from *gsb*-*int*-Prd and *gsb*-*int*-Pax3, respectively.

The *gsb-*Prd and *gsb-*Pax3 constructs were injected together with pUChspΔ2-3 helper plasmid into *ry^506^* embryos and *ry* ^+^ transformants were selected.

### Immunostaining and *in situ* hybridization of embryos

Embryo collection, fixation, and immunostaining were carried out as described [28]. Polyclonal antibodies against Prd (1∶500) [28] Gsb, and Gsbn (1∶1000) [9], monoclonal antibody against Wg (1∶100) [29], and monoclonal antibody BP102 (1∶50), which reveals the patterns of the longitudinal and commissural axons in the CNS [11], have been described. Polyclonal anti-ß-galactosidase antibody (1∶1000) was obtained from Cappell.

*In situ* hybridization with digoxigenin-labeled *Pax3* cDNA was performed essentially as described [25].

### Cuticle preparation

Embryos were collected and allowed to develop for 24 h at 25°C before cuticles were prepared as described [1].

### Fly strains and rescue experiments

Three *gsb* alleles were used in this work: *Df(2R)IIX62*, a *gsb* null allele that deletes *gsb*, *gsbn*, and five additional genes [17], [30]; *gsb^525^*, a strong hypomorphic allele in which the first amino acid of the homeodomain is converted to a stop codon [11]; and *gsb^P1155^*, a hypomorphic allele with a P-element inserted into the *gsb* promoter region [11]. To rescue the cuticle, CNS, viability, and male fertility functions of *gsb* by the transgenes, we used the following fly stocks: (1) *Df(2R)IIX62/SM1*, (2) *gsb^525^/SM1*, (3) *gsb^P1155^/SM1*, (4) *Df(2R)IIX62/SM1*; *gsb-res*, (5) *gsb^525^/SM1*; *gsb-res*, (6) *Df(2R)IIX62/SM1*; *gsb-*Prd, (7) *gsb^525^/SM1*; *gsb-Prd*, (8) *Df(2R)IIX62/SM1*; *gsb-*Pax3, and (9) *gsb^525^/SM1*; *gsb-*Pax3.
